The article "An Image Fusion Algorithm Based on Improved RGF and Visual Saliency Map" was retracted in 2023. Reasons: signs of a paper mill; suspected computer-generated content; unreliable results or conclusions; concerns about the data.

# An Image Fusion Algorithm Based on Improved RGF and Visual Saliency Map

**DOI:** 10.1155/2022/1693531

**Published:** 2022-08-25

**Authors:** Yang Li, Haitao Yang, Yuge Gao

**Affiliations:** Center for Space Security Studies, University of Aerospace Engineering, Beijing, China

## Abstract

To solve the artifact problem in fused images and the lack of enough generalization under different scenarios of existing fusion algorithms, the paper proposes an image fusion algorithm based on improved RGF and visual saliency map to realize fusion for infrared and visible light images and a multimode medical image. Firstly, the paper uses RGF (rolling guidance filter) and Gaussian filter to decompose the image into the base layer, interlayer, and detail layer by a different scale. Secondly, the paper obtains a visual weight map by the calculation of the source image and uses the guided filter to better guide the base layer fusion. Then, it realizes the interlayer fusion through maximum local variance and realizes the detail layer fusion through the maximum absolute value of the pixel. Finally, it obtains the fused image through weight fusion. The experiment demonstrates that the proposed method shows better comprehensive performance and obtains better results in fusion for infrared and visible light images and medical images compared to the contrast method.

## 1. Introduction

As an image enhancement technology, image fusion basically aims to form a fused image that is more useful for human vision or subsequent image processing by superimposing and complementing all information of two or more images under the same scenario for different sensors or different positions, time, and illumination. The process shall follow three basic rules: firstly, the fused image must retain distinct features of the source image. Secondly, artificial information cannot be added in the fusion process. Thirdly, the valueless information (e.g., noise) shall be restrained as much as possible.

Among medical images, the multimode image can provide various types of information, of which importance on the clinical diagnosis increases continuously. Based on different imaging mechanisms, the multimode medical image provides different types of organizational information. For example, CT (computed tomography) provides information on the dense structure (e.g., skeleton and implantation material), whereas MR-T2 (T2-weighted magnetic resonance imaging) indicates high-resolution anatomical information (e.g., soft tissue). To obtain enough information for accurate diagnosis, doctors often need to make sequence analyses for captured medical images under different modes. In many cases, such a separated diagnosis mode is not convenient. An effective method of solving the problem is medical image fusion, which aims to generate a combined image and integrate complementary information in different forms of medical images.

The article "An Image Fusion Algorithm Based on Improved RGF and Visual Saliency Map" was retracted in 2023. Reasons: signs of a paper mill; suspected computer-generated content; unreliable results or conclusions; concerns about the data.

With the rapid development of image technology in theory and application, how to improve information content in the fused image and how to improve the speed of fusion algorithm and generalization under different application scenarios are widely studied. Based on Laplacian Pyramid transform [1] and wavelet transforms [2], the early multiscale fusion method combines with different fusion rules or optimizes the decomposition method to improve the fusion effect or speed. However, the algorithm based on the above two methods has theoretical defects, i.e., the Pyramid decomposition-based method has no translation invariance but excessive redundant information, whereas the wavelet variation-based method has no translation invariance and few directions of decomposition. Therefore, the derived algorithm from the above methods obtains an unclear target edge of the fused image and a bad overall effect. Although the NSCT (nonsubsampled contourlet)- [3] and NSST (nonsubsampled shearlet transform)-based [4] methods can overcome the above problems, realize good direction selection and translation invariance, generate less redundant information and more details in the fused image when decomposing the image, the methods cannot ensure spatial consistency in the fusion process and may result in an artifact in the fused image and noise because of the algorithm.

For the problems and defects of the above algorithm, the paper proposes the RGF-based improvement method for decomposing the source image on the basis of a conventional algorithm, and it designs a new fusion algorithm in combination with the maximum local variance, the maximum absolute value of the pixel, and a visual saliency map. Through the experimental verification of visual light and infrared image fusion and medical image fusion, the proposed algorithm indicates a better fusion effect, clearer edge in the fused image, higher illumination of the infrared target, more complete background information of visible light in the fused image, and better generalization under different scenarios compared to the classical algorithm.

## 2. Related Algorithm Research

### 2.1. Guided Filter and Rolling Guidance Filter (RGF)

He et al [5] proposed the guided filter in 2010, which attracted wide attention because of its salient boundary effect, good gradient retention, and low linear complexity. Compared to other filters, the method can enhance detailed information and the overall feature of an image while retaining good image edge information.

The article "An Image Fusion Algorithm Based on Improved RGF and Visual Saliency Map" was retracted in 2023. Reasons: signs of a paper mill; suspected computer-generated content; unreliable results or conclusions; concerns about the data.

The basic principle of the guided filter can be explained as follows: if the input image is *p*, the output image is *q*, and the guided image is *I*, then the output image *q* in the window *ω*_*k*_ with the center of *k* can be expressed as

(1) $$\begin{array}{c} q_{i}=a_{k}I_{i}+b_{k},\;\forall i\in \omega_{k}, \end{array}$$

where *i* & *k* are pixel coordinates, *a*_*k*_ & *b*_*k*_ are linear constants in the window, and *ω*_*k*_ is the square window with a size of (2*r*+1)(2*r*+1). It can be seen that ∇*q*=*a*∇**I** is true and ensures edge consistency between the output image *q* and the guided image *I*.

The constants *a*_*k*_ and *b*_*k*_ can be calculated by minimizing the square error between the input image *p* and the output image *q*:

(2) $$\begin{array}{c} E\left(a_{k},b_{k}\right)=\sum_{i\in \omega_{k}}\left[{\left(a_{k}I_{k}+b_{k}-p_{i}\right)}^{2}+\varepsilon a_{k}^{2}\right], \end{array}$$

where *ε* is the regularization parameter that can avoid too large a coefficient. Then, *a*_*k*_ and *b*_*k*_ can be calculated as follows:

(3) $$\begin{array}{c} a_{k}=\frac{\left(1/\left|\omega \right|\right)\sum_{i\in \omega_{k}}I_{i}p_{i}-\mu_{k}\bar{p_{k}}}{\sigma_{k}^{2}+\varepsilon },\\ b_{k}=\bar{p_{k}}-a_{k}\mu_{k}, \end{array}$$

where *μ*_*k*_ and $\bar{p_{k}}$ are the mean values of *I* and *p* in the window *ω*_*k*_, *σ*_*k*_^2^ is the variance of *I* in the window *ω*_*k*_, and |*ω*| is the pixel of window *ω*_*k*_.

It is given that the guided image *I* has a linear correlation in the window *ω*_*k*_, and the window includes all pixel points *p*_*i*_, so that the value of the output image will vary with the transform of the window *ω*_*k*_. Then, the final filter output *q*_*i*_ can be expressed as follows:

(4) $$\begin{array}{c} q_{i}=\frac{1}{\left|\omega \right|}\sum_{i\in \omega_{k}}\left(a_{k}I_{k}+b_{k}\right)=\bar{a_{i}}I_{i}+\bar{b_{i}}. \end{array}$$

The final guided filter can be expressed as follows:

(5) $$\begin{array}{c} q=G_{r,\varepsilon }\left(I,p\right), \end{array}$$

where *G* is the guided filter, and *r*, *ε* are the sizes of the filter window and structural erasing scale.

RGF [6] (rolling guidance filter) is an iteration method of combining the guided filter with other filters. It can obtain the outline of the object when filtering an image. Compared to other filters, RGF can avoid the loss of outline and boundary when erasing the texture structure or area details.  Figure 1 shows the key idea of iteratively processing an image by RGF.

#### 2.1.1. Small Structure Removal

The paper, firstly, erases the edge of the source image *J* to obtain *J*_1_. Then, it considers the source image *J* as the guided image and uses the guided filter for *J*_1_ to recover the edge and obtains *J*_2_. Compared to *J*_1_, *J*_2_ has a clearer edge, and it loses some detail texture. The paper repeats the above steps and gradually increases the scale of erasing details to obtain the filtering results of a different scale.

The article "An Image Fusion Algorithm Based on Improved RGF and Visual Saliency Map" was retracted in 2023. Reasons: signs of a paper mill; suspected computer-generated content; unreliable results or conclusions; concerns about the data.

The materials and methods section should contain sufficient details, so that all procedures can be repeated. It may be divided into headed subsections if several methods are described.

### 2.2. Visual Saliency Analysis

Visual saliency is an expression method of extracting salient points or areas in an image in a visual form by simulating human eyes, observing various features under different scenarios and generating related strong and weak stimulation. The first step of obtaining a visual saliency map is to get its high-pass image. The basic method is to use the difference between the mean filtering result and median filtering result of the source image to obtain the corresponding high-pass image, with the expression given as follows:

(6) $$\begin{array}{c} H_{n}\left(x,y\right)=\text{Average filter}\left(x,y,\mu_{n}\right)-\text{Median filter}\left(x,y,\rho_{n}\right),\\ n=1,2, \end{array}$$

where (*x*, *y*) is the pixel coordinate of the source image in the corresponding position, and *μ*_*n*_ and *ρ*_*n*_ are the sizes of the mean filtering window and median filtering window.

The visual saliency map of two source images can be obtained by the smooth operation of the Gaussian filter based on the high-pass image, with the expression given as follows:

(7) $$\begin{array}{c} S_{n}=\text{Gaussian filter }\left(H_{n},r_{g},\sigma_{g}\right), \end{array}$$

where (2*r*_*g*_+1)(2*r*_*g*_+1) is the window size of the Gaussian filter, *σ*_*g*_ is the standard deviation of the filter, and **S**_*n*_ is the obtained visual saliency map.

## 3. Fusion Algorithm Design

### 3.1. RGF-Based Image Decomposition Algorithm

As a filter with good dimensional perception and edge retention characteristic, RGF is widely used for extracting the edge outline and denoising the image. RGF consists of structural erasure and edge recovery. The first step is to eliminate a small structure with the filter, in which a Gaussian filter and median filter can be used. The proposed improved RGF structure consists of a guided filter and a mean filter. If the mean filter is used for structural erasure, it indicates high mean filtering efficiency, simple and fast computation, and the stable erasure of information in the spatial scale. As a result, the extracted features of different scales are separated more thoroughly. If the input image is I, the obtained output filtering image *G* can be expressed as follows:

(8) $$\begin{array}{c} G=\text{Average }\left(I,\sigma_{s}\right), \end{array}$$

where *σ*_*s*_ is the scale parameter. Theoretically, the step can erase the structure with a smaller spatial scale than *σ*_*s*_. Secondly, the paper uses the guided filter, recursive bilateral filter, or bilateral filter for edge recovery. Although the bilateral filter has a better edge retention effect, it requires calculating the spatial filtering kernel function and the grey filtering kernel function simultaneously, of which the frequency response has a correlation with the input image. Hence, the bilateral filter is not applicable here because it is nonlinear and takes a long execution time. The paper selects the guided filter for the second step of edge recovery. If the iterative recovery for edge is made for the image J^t^, then the obtained iterative image *J*^t + 1^ can be expressed as follows:

(9) $$\begin{array}{c} J^{t+1}=\text{Guided Filter }\left(J^{t},I,\sigma_{s},\sigma_{r}^{2}\right), \end{array}$$

where *I* is the guided image. The paper selects the source image as a guided image to recover the edge structure to the largest extent. *σ*_*r*_ is the distance weight, and *σ*_*s*_ is the scale parameter.

The article "An Image Fusion Algorithm Based on Improved RGF and Visual Saliency Map" was retracted in 2023. Reasons: signs of a paper mill; suspected computer-generated content; unreliable results or conclusions; concerns about the data.

The above formula can be expressed as follows:

(10) $$\begin{array}{c} u=\text{RGF }\left(I,\sigma_{s},\sigma_{r},T\right), \end{array}$$

where the number of iterations is set to *T*=4, and *u* is the output image.

The front four images show the results of iterative smoothness with RGF (mean value—guided filter), and the final image shows the fuzzy result of the Gaussian filter. It can be seen that the edge structure is erased by different scales during iterative smoothness with RGF (mean value—guided filter). The change in the image is shown in Figure 2. Compared to the first image, the wall detail, small bicycle in the far distance, and texture on the ground are erased in the second image. Compared to the second image, the outline of the small structure is vague, and the edge of some large structures is dissolved in the third image. The fourth image includes the edges of the large structure and target. The iterative results accommodate the demand hereof.

Figure 3 shows the multiscale decomposition results of the extracted image from different iterative results. The image is decomposed into four layers here. The final image shows the Gaussian blur result of the source image, which is considered the base layer. The base layer generally includes the overall contrast ratio and grey distribution in the image and erases the edge detail information in the source image. The paper considers the 5^th^ layer as the base layer, which can be obtained directly through Gaussian filter processing to include rough grey distribution and an overall contrast ratio of the image. Compared to the method of obtaining the base layer through continuous iteration, direct processing for the source image is simpler, faster, and better. The detail layer and interlayer are obtained from the front four images, where *J*_1_*J*_2_ correspond to the portions with small structure and *J*_3_*J*_4_ correspond to the portions with large structure. Different scale of information is decomposed to different images.

The article "An Image Fusion Algorithm Based on Improved RGF and Visual Saliency Map" was retracted in 2023. Reasons: signs of a paper mill; suspected computer-generated content; unreliable results or conclusions; concerns about the data.

Image decomposition can be expressed as follows:

(11) $$\begin{array}{c} u^{j}=\text{RGF}\left(u^{j-1},\sigma_{s}^{j-1},\sigma_{r},T\right),\;\left(j=1,\ldots ,N-1\right), \end{array}$$

(12) $$\begin{array}{c} d^{j}=u^{j-1}-u^{j},\;\left(j=1,\ldots ,N-1\right), \end{array}$$

(13) $$\begin{array}{c} u^{j}=\text{Gaussian}\left(u^{j-1},\sigma_{s}^{j-1}\right),\;\left(j=N\right), \end{array}$$

(14) $$\begin{array}{c} d^{j}=u^{j-1}-u^{j},\;\left(j=N\right), \end{array}$$

where formulas (11) and (12) are the iterative expressions of the detail layer and interlayer, *u*^*j*^ is the image in the *j*^th^ iteration, *d*^*j*^ is the image in the *j*^th^ decomposition, and *N* is the number of decomposed layers. Formulas (13) and (14) are used for solving the base layer. With the above formulas, the paper decomposes the source image into a base layer, interlayer, and detail layer.

### 3.2. Design of Fusion Method

Figure 4 shows the overall design of the proposed fusion method. Firstly, the paper decomposes the image into the base layer, interlayer, and detail layer through MSD (multiscale decomposition) to include the different scale information of the image. Secondly, the paper uses the processed visual saliency map by the guided filter to guide the base layer fusion, uses the maximum local variance to guide interlayer fusion, and uses the maximum absolute value of the pixel to guide the detail layer fusion.

### 3.3. Interlayer and Detail Layer Fusion

The detail layer is separated from the source image and includes small structure and texture characteristics, of which the fusion effect directly influences the fusion result. The paper selects *L*1*L*2 as detail layers for fusion through the maximum absolute value of the pixel. The method is generally used for the fusion of high-frequency portions in the image. If the values of a pixel pair on the detail layer of the source image are *d*_1_ and *d*_2_, then the weight of the processed point through the maximum absolute value of pixel *W* is as follows:

(15) $$\begin{array}{c} W^{j}=\left\{\begin{array}{cc} 1, & \left|d_{1}^{j}\right|>\left|d_{2}^{j}\right|\\ 0, & \text{otherwise} \end{array}\;\left(j=1,2,\ldots ,N\right)\right). \end{array}$$

Then, the detail layer *M*^*j*^ can be expressed as follows:

(16) $$\begin{array}{c} M^{j}=W_{d}^{j}d_{1}^{j}+\left(1-W_{d}^{j}\right)d_{2}^{j}\;\left(j=1,2\right). \end{array}$$

The information structure in the interlayer is larger than the detail layer and smaller than the base layer in scale, which includes the edge and outline of the large structure. For such information, the paper selects the fusion pixel through maximum local variance. The pixel region with a large local variance represents a larger information content, so that more salient characteristics in the source image can be retained in the fusion result. If the local region is (2*d*+1)(2*d*+1) and the number of local pixel points is *n*, then the local variance can be expressed as follows:

(17) $$\begin{array}{c} V\left(x\right)=\sqrt{\frac{1}{n-1}\sum_{x=1}^{n}{\left(i\left(x\right)-u\right)}^{2}},\\ u=\frac{1}{n}\sum_{x=1}^{n}i\left(x\right)n. \end{array}$$

In the local variance map of the above two images, if the weight of the pixel point with large variance is 1 and the weight of the pixel point with small variance is 0, then the fused image *M*^*j*^ on the interlayer is expressed as follows:

(18) $$\begin{array}{c} W^{j}=\left\{\begin{array}{cc} 1, & V_{1}^{j}\left(x\right)>V_{2}^{j}\left(x\right)\\ 0, & \text{otherwise} \end{array}\;\left(j=3,4\right)\right),\\ M^{j}=W_{d}^{j}d_{1}^{j}+\left(1-W_{d}^{j}\right)d_{2}^{j}\;\left(j=3,4\right). \end{array}$$

The article "An Image Fusion Algorithm Based on Improved RGF and Visual Saliency Map" was retracted in 2023. Reasons: signs of a paper mill; suspected computer-generated content; unreliable results or conclusions; concerns about the data.

### 3.4. Base Layer Fusion

In the decomposition method, the obtained base layer includes grey distribution and a contrast ratio of the source image to regulate the overall visual perception of the fused image. The simple fusion rule is generally selected during the fusion. On the one hand, it can improve the fusion speed. On the other hand, the low-frequency information is not useful and cannot be processed by a complex method. However, these simple fusion rules with representative “averaging” fusion rule have low utilization for low-frequency information and neglect the difference of low-frequency information in different source images, resulting in a decrease in contrast ratio in the fused image and a bad fusion effect.

For the above problem, the paper proposes an adaptive fusion method for a visual saliency map under the guidance of a guided filter to realize the base layer fusion. The visual saliency analysis is widely used in the field of computer vision, which can reflect the salient characteristics of the image and recognize visual structure and object with salient perception in the image different from adjacent regions. The paper uses the method of Literature [7] to build VSM, which considers the comparison between a pixel point and an adjacent pixel point as the definition of pixel saliency. If *I*_*p*_ is the intensity value of a pixel point *p* in the image, then the visual saliency *V*(*p*) of the pixel *p* is defined as follows:

(19) $$\begin{array}{c} V\left(p\right)=\left|I_{p}-I_{1}\right|+\left|I_{p}-I_{2}\right|+\cdots +\left|I_{p}-I_{N}\right|, \end{array}$$

where *N* is the total number of pixel points in the image *I*. If two pixels have the same intensity values, then they have the same saliency. The larger the intensity value, the stronger the saliency. The formula can be updated as follows:

(20) $$\begin{array}{c} V\left(p\right)=\sum_{j=0}^{L-1}M_{j}\left|I_{p}-I_{j}\right|, \end{array}$$

where *j* is the different pixel intensity, *M* is the number of pixels with intensity *j*, and *L* is the number of grey levels (total 256). The weight map from direct calculation indicates a bad fusion effect for the base layer. The paper uses the guided filter and selects the original image *I* as the guided image for filtering the weight map.

(21) $$\begin{array}{c} V^{\prime }=\text{Guided Filter}\left(V,I,\sigma_{s},\sigma_{r}^{2}\right). \end{array}$$

The paper uses an adaptive “mean value” rule during fusion. The formula is as follows:

(22) $$\begin{array}{c} W_{b}=0.5+\frac{V_{1}^{\prime }-V_{2}^{\prime }}{2}, \end{array}$$

where *V*1 and *V*2 are processed visual saliency maps by the guided filter, respectively. If *V*_1_=*V*_2_, then *W*_*b*_=0.5. It is the weight of the mean value at the point. If *V*_1_ > *V*_2_, then the weight *W*_*b*_ will increase, and more information in the fusion result will be obtained from *V*_1_. Otherwise, the weight will decrease and more information in the fusion result will be obtained from *V*_2_. Then, the fused result from the weighting average can be expressed as follows:

(23) $$\begin{array}{c} B_{F}=W_{b}B_{1}+\left(1-W_{b}\right)B_{2}. \end{array}$$

The article "An Image Fusion Algorithm Based on Improved RGF and Visual Saliency Map" was retracted in 2023. Reasons: signs of a paper mill; suspected computer-generated content; unreliable results or conclusions; concerns about the data.

## 4. Experiment and Result Analysis

### 4.1. Experimental Environment and Design

In the experiment, the hardware configuration is a PC with Intel (R) Core (TM) i5-9600k 3.7 GHz CPU and NVIDIA GeForce RTX 1080ti GPU, and the software configuration is MATALB 2021b.

The paper selects 15 pairs of infrared and visible light images from the TNO dataset, which can verify the validity and advancement of the fusion algorithm because the image subjects include character, carrier, building, and hidden target. Besides, the paper selects CT and MRI image pairs to verify the generalization of the algorithm.

The experiment compares the proposed algorithm with five classical algorithms, i.e., RP (ratio pyramid) transform-based method, CVT (curvelet) variation-based method [8, 9], curvelet_sr transform-based method [10], CBF (cross bilateral filter)-based method [11], and NSCT transform-based method [12].

### 4.2. Analysis of Experimental Results for Infrared and Visible Light Image Fusion

#### 4.2.1. Comparison of Subjective Results

Figure 5 shows a parallel comparison of fusion results for infrared and visible light images under different scenarios, where Figures 5 (1) and (2) show the infrared and visible light images, and Figures 5 (3) to (8) show algorithm comparison. To conveniently show algorithm results, the paper selects and magnifies some portions and the above images.

It can be concluded through intuitive observation that the fusion results of the CBF algorithm include much meaningless noise, bad edge fusion effect, and more serious distortion of fused images. For CVT and CVTSR algorithms, the infrared target is generally reflected. The fused image includes a small number of noises. The CVT algorithm results in a serious artifact, whereas the CVTSR algorithm results in a slight artifact and a relatively low contrast ratio. The NSCT algorithm indicates a good contrast ratio, more complete information of visible light, but low illumination of the infrared target, and a nonsalient target. The RP algorithm indicates relatively high illumination of fusion, fluorescent characteristic, salient infrared information, however, it results in the serious erasure of visible light information, and a serious loss of edge details. The proposed algorithm can realize better fusion for the information of infrared and visible light images, avoid artifacts at the edge boundary, indicate salient infrared characteristics, and retain the good details of visible light and good visual effect as a whole. Therefore, the method can realize a better fusion effect for infrared and visible light images compared to contrast algorithms.

#### 4.2.2. Comparison of Objective Results

The paper evaluates the fusion results of the proposed algorithm through 9 indexes, i.e., CC (correlation coefficient) [13], EN (entropy) [14], SSIM (structural similarity) [15], Qab/*f* [16], VIF (visual information fidelity) [17], SCD (sum of correlation difference) [18], MS-SSIM (multilevel structural similarity) [7], MI (mutual information) [19], and SD (standard deviation) [20].

To avoid the contingency of a single image, the paper considers the mean values of evaluation indexes of 14 images from Figure 5 as contrast indexes, implements visualization for data in Figure 6, and marks optimal results in red. It can be seen from Table 1 and Figure 6 that the paper obtains optimal and suboptimal values from CC, SSIM, SCD, MS-SSIM, and MI. It indicates that the proposed algorithm has a good correlation with the source image and retains more useful information. The best values from EN, VIF, Qab/*f*, and SCD that the fusion results of the proposed algorithm indicate a better visual effect and larger information content.

The article "An Image Fusion Algorithm Based on Improved RGF and Visual Saliency Map" was retracted in 2023. Reasons: signs of a paper mill; suspected computer-generated content; unreliable results or conclusions; concerns about the data.

To sum up, the analysis of objective data demonstrates the superiority of the proposed algorithm.

### 4.3. Analysis of Experimental Results for Medical Image Fusion

To verify the generalization and application effect of the proposed algorithm in the medical image, the paper selects four groups of multimode brain lesion images with the size of 256 × 256 for the contrast experiment. Figures 7 (1) and (2) show the multimode images. Figures 7 (3) to (8) show result comparisons of different algorithms.

#### 4.3.1. Comparison of Subjective Results

As shown in Figure 7, the CBF method indicates a good contrast ratio of fusion results but serious artifact and noise. CVT and CVTSR methods indicate the overall dark image and vague edge structure. The NSCT method indicates overall vague fusion result, which is not beneficial to the human eye recognition and subsequent computer processing. The RP method indicates overall excessive illumination of the fusion result and incomplete image information. Compared to the fusion effect hereof, the proposed algorithm indicates a good contrast ratio and detailed information, integrates different information of multimode images, and realizes the purpose of image fusion well.

#### 4.3.2. Comparison of Objective Results

Table 2 shows the mean values of results for four groups of multimode medical image fusion, where bold values are optimal, and visual processing is shown in Figure 8. It can be seen that the proposed algorithm obtains optimal or suboptimal values among all contrast indexes. According to all subjective and objective evaluations, the proposed algorithm can realize the optimal fusion effect in multimodel medical images, integrate information from the source image, and benefit subsequent human eye judgment or computer processing compared to contrast algorithms.

## 5. Conclusions

The paper proposes an image fusion algorithm based on improved RGF and visual saliency map. Firstly, the paper uses RGF to decompose the image into the base layer, interlayer, and detail layer at different scales. Secondly, the paper obtains a visual weight map through the calculation of the source image and uses the guided filter to better guide the base layer fusion. Then, it realizes the interlayer fusion through maximum local variance and realizes the detail layer fusion through the maximum absolute value of the pixel. Finally, it obtains the fused image through weight fusion. The experiment uses the infrared and visible light image pair and multimode medical image pair to compare and verify the proposed algorithm. The experimental results indicate that the proposed method is better than the contrast algorithm in subjective effect and objective evaluation. Besides, the fused image with better details, edge, and texture retention capacity and good overall contrast ratio can be obtained with the proposed algorithm.

The article "An Image Fusion Algorithm Based on Improved RGF and Visual Saliency Map" was retracted in 2023. Reasons: signs of a paper mill; suspected computer-generated content; unreliable results or conclusions; concerns about the data.

## Figures and Tables

**Figure 1:** RGF diagram.

**Figure 2:** Iterative smoothness with RGF (mean value—guided filter).

**Figure 3:** Iterative decomposition with RGF (mean value—guided filter).

**Figure 4:** The proposed decomposition method.

**Figure 5:** Comparison of the fusion results from different methods on the source images.

**Figure 6:** Comparison of the fusion results from different methods on the source images.

**Figure 7:** Comparison of the fusion results from different methods on the source images.

**Figure 8:** Comparison of the fusion results from different methods on the source images.

**Table 1:** Different fusion methods are compared quantitatively, and the best fusion results are highlighted in bold.

Indexes	Methods					
	rp	Curvelet	Curvelet_sr	CBF	NSCT	Proposed
CC	0.3576	0.4694	0.4824	0.3656	0.4830	**0.5245**

EN	7.5463	7.5871	7.5863	7.6432	7.6142	**7.6970**

SSIM	0.6172	0.6617	0.6690	0.5136	0.7049	**0.7310**

Qabf	0.2387	0.3333	0.3228	0.2922	**0.3727**	0.3493

VIF	0.3059	0.3684	0.3513	0.3293	0.4215	**0.4637**

SCD	1.0800	1.3965	1.4432	1.1196	1.4535	**1.4569**

MSSSIM	0.6147	0.6707	0.6906	0.4963	0.7190	**0.7388**

MI	1.2008	1.2772	1.3150	**1.5968**	1.3481	1.5894

SD	9.5468	9.9837	10.0149	9.9406	9.9828	**10.0604**

**Table 2:** Different fusion methods are compared quantitatively, and the best fusion results are highlighted in bold.

Methods	Indexes					
	rp	Curvelet	Curvelet_sr	CBF	NSCT	Proposed
CC	0.7504	0.7093	0.7401	0.7533	0.7250	**0.7807**

EN	6.9483	7.5573	7.5092	7.1027	7.5090	**7.6053**

SSIM	0.6789	0.6990	0.7107	0.7647	0.7778	**0.8214**

Qabf	0.3325	0.3995	0.4071	0.4887	0.4891	**0.5009**

VIF	0.5328	0.4246	0.4103	**0.6002**	0.5038	0.5912

SCD	0.6646	0.6468	0.6991	0.7658	0.7557	**0.8521**

MSSSIM	0.7305	0.7715	0.7865	0.8007	0.8378	**0.8429**

MI	3.0110	2.5652	2.6563	2.8093	2.8856	**3.2338**

SD	9.9432	10.1073	10.1456	10.3472	10.1509	**10.4893**

## Data Availability

The basis of data from TNO_Image_Fusion_Dataset is used this article, and the details can be found in https://figshare.com/articles/TN_Image_Fusion_Dataset/1008029.

The article "An Image Fusion Algorithm Based on Improved RGF and Visual Saliency Map" was retracted in 2023. Reasons: signs of a paper mill; suspected computer-generated content; unreliable results or conclusions; concerns about the data.

## References

[1] Burt P. J., Adelson E. H., Fischler M. A., Firschein O. (1987). The laplacian pyramid as a compact image code. *Readings in Computer Vision: Issues, Problem, Principles, and Paradigms*.

[2] Pajares G., de la Cruz J. M. (2004). A wavelet-based image fusion tutorial. *Pattern Recognition*.

[3] Chen M. S. (2016). Image fusion of visual and infrared images based on NSCT and compressed sensing. *Journal of Image and Graphics*.

[4] Zhang B. H., Lu X. Q., Pei H. Q., Zhao Y. (2015). A fusion algorithm for infrared and visible images based on saliency analysis and non-subsampled shearlet transform. *Infrared Physics & Technology*.

[5] He K., Jian S., Tang X. (2010). *Guided Image filtering*.

[6] Zhang Q., Shen X., Xu L., Jia J. (2014). *Rolling Guidance Filter*.

[7] Chen M. J., Bovik A. C. (2010). Fast structural similarity index algorithm. *Journal of Real-Time Image Processing*.

[8] Lewis J. J., O’Callaghan R. J., Nikolov S G, Nikolov S. G., Bull D. R., Canagarajah N. (2007). Pixel- and region-based image fusion with complex wavelets. *Information Fusion*.

[9] Nencini F., Garzelli A., Baronti S., Alparone L. (2007). Remote sensing image fusion using the curvelet transform. *Information Fusion*.

[10] Li S., Yang B., Hu J. (2011). Performance comparison of different multi-resolution transforms for image fusion. *Information Fusion*.

[11] Shreyamsha Kumar B. K. (2015). Image fusion based on pixel significance using cross bilateral filter. *Signal, Image and Video Processing*.

[12] Zhang Q., Guo B.-L. (2009). Multifocus image fusion using the nonsubsampled contourlet transform. *Signal Processing*.

[13] Edelmann D., Móri T. F., Székely G. J. (2021). On relationships between the pearson and the distance correlation coefficients. *Statistics & Probability Letters*.

[14] Bulanon D. M., Burks T., Alchanatis V. (2009). Image fusion of visible and thermal images for fruit detection. *Biosystems Engineering*.

[15] Wang Z., Bovik A. C., Sheikh H. R., Simoncelli E. P. (2004). Image quality assessment: from error visibility to structural similarity. *IEEE Transactions on Image Processing*.

[16] Petrovic V., Xydeas C. (2000). Objective image fusion performance measure. *Electronic Letters*.

[17] Bovik H. (2006). Image information and visual quality. *Ieee Transactions on Image Processing a Publication of the Ieee Signal Processing Society*.

[18] Pack A. I. (2022). AEÜ—international journal of electronics and communications. *International Journal of Electronics and Communications*.

[19] Qu G., Zhang D., Yan P. (2002). Information measure for performance of image fusion. *Electronics Letters*.

[20] Rao Y.-J. (1997). In-fibre bragg grating sensors. *Measurement Science and Technology*.

